# Identification of Key Gene Targets for Periodontitis Treatment by Bioinformatics Analysis

**DOI:** 10.1155/2022/7992981

**Published:** 2022-09-29

**Authors:** Ying Jin, Ye Wang, Xiaoping Lin

**Affiliations:** Department of Stomatology, Shengjing Hospital of China Medical University, Shenyang, Liaoning, China

## Abstract

**Background:**

Periodontitis is considered to be the leading cause of tooth loss in adults, and it interacts with some serious systemic diseases. Periodontal basic therapy is the cornerstone of periodontal disease treatment and long-term maintenance and has a positive impact on the treatment of systemic diseases.

**Aim:**

To explore the potential gene targets of periodontitis therapies by bioinformatics method.

**Methods:**

We analyzed the expression database (GSE6751) downloaded from the Gene Expression Omnibus (GEO) with weighted gene coexpression network analysis (WGCNA) to confirm the functional gene modules. Pathway enrichment network analyses the key genes in functional modules and verified the candidate genes from the samples in peripheral blood sources of GSE43525. Moreover, we confirmed the expression of target protein in the periodontal tissues of experimental periodontitis-afflicted mice using western blotting.

**Results:**

The functional gene modules were found to have biological processes, and *ARRB2*, *BIRC3*, *CD14*, *DYNLL1*, *FCER1G*, *FCGR1A*, *FCGR2B*, *FGR*, *HCK*, and *PRKCD* were screened as candidates' genes in functional modules. The 921 DEG from GSE43525 and 418 DEG is from the green module of GSE6751 and identified *AMICA1*, *KDELR1*, *DHRS7B*, *LMNB1*, *CTSA*, *S100A12*, and *FCGR1A* as target genes. Finally, FCGR1A (CD64) was confirmed as the key gene that affects periodontal treatment. Western blot analysis showed an increasing trend in the expression level of FCGR1A protein in the periodontal tissues of experimental periodontitis mice compared to normal mice.

**Conclusions:**

FCGR1A (CD64) may be a key gene target for periodontal therapy in patients with periodontitis and other systemic diseases.

## 1. Introduction

Periodontal disease results from an imbalance in the local immune microenvironment of periodontal tissues. Pathogens invade periodontal tissues, including tissues surrounding dental implants, stimulating the body's immune system and leading to the infiltration of chemokines and inflammatory cells, which triggers the destruction of periodontal supporting tissues [1]. Periodontal disease is the leading cause of tooth loss in adults, with a high incidence worldwide. Furthermore, increasing evidence demonstrates a correlation between periodontal disease and systemic diseases, such as diabetes, autoimmune inflammatory diseases, atherosclerosis, and vascular diseases [2–6].

As the initial stage of periodontal therapy, periodontal basic therapy can slow or block the development of periodontal inflammation over time. Several studies have shown that local periodontal nonsurgical treatment significantly affects gene expression patterns in peripheral blood mononuclear cells. Currently, at least 65 genes are thought to be associated with periodontitis [7]. This diversity in gene expression patterns is likely to affect the prognosis of patients with periodontitis associated with systemic disease [8].

The discovery and development of periodontitis in systemic diseases are complex systematic biological processes across various functional networks. The application of bioinformatics methods such as systematic description, screening of important information, and high-throughput research and data analysis can identify complex functional networks. In the published literature, weighted gene coexpression network analysis (WGCNA) was used to analyze potential gene modules that function in gene expression data [9]. The WGCNA selects weighting coefficients to obtain results most consistent with the scale-free network distribution. Comprehensive data analysis will help clinicians better understand the function of genes and their relationship with disease [10].

This study analyzed the effects of comprehensive periodontal therapy on gene expression in peripheral blood mononuclear cells of patients with periodontitis using the standard WGCNA program. To dissect the relationship between gene modules and the comprehensive treatment of periodontitis, we screened candidate genes that affect the treatment of periodontitis and identified key biomarkers related to periodontal diseases associated with systemic diseases.

## 2. Materials and Methods

### 2.1. Data Acquisition

“Periodontal therapy,” “peripheral blood mononuclear cells,” and “periodontal disease” were used as key words to search gene expression datasets related to periodontal disease in public Gene Expression Omnibus (GEO), a comprehensive gene expression database supported by the National Center for Biotechnology Information (NCBI) of the American National Library of Medicine (NLM). The series matrix files and data tables of the microarray platform from GSE6751 (https://www.ncbi.nlm.nih.gov/geo/query/acc.cgi?acc=GSE6751) and GSE43525 (https://www.ncbi.nlm.nih.gov/geo/query/acc.cgi?acc=GSE43525) were downloaded from the GEO, and GSE6751 consists of 59 blood samples taken from 15 separate periodontitis patients with comprehensive treatment at four different time points: 15 samples taken one week prior to periodontal therapy, 14 samples taken at treatment initiation (baseline), 15 samples taken six weeks postbaseline, and 15 samples taken 10 weeks postbaseline. GSE43525 contains nine transcriptome data samples (five blood samples from patients with refractory periodontitis and four blood samples from healthy patients); these data were used for subsequent model validation.

### 2.2. Coexpression Network Construction by WGCNA

We constructed a weighted coexpression gene network of GSE6751 gene data using the WGCNA-R package (R project version 4.0.0). We identified coexpressed gene modules to explore phenotypes and core genes in the gene network. The top 5000 genes were selected using this algorithm for further analysis. WCGNA instruments were used to frame the network in the form of a soft threshold *β*. In this study, *β* was estimated according to scale-free criteria, and the topological overlap matrix (TOM) was transformed from the degree of adjacency among the genes. Based on the weighted correlation coefficient, genes were classified according to their expression patterns, and genes with similar patterns were grouped into one module. According to the dissimilarity matrix, a hierarchical clustering tree diagram was estimated for the genes, and the gene modules were calculated using the dynamic branch cutting method.

### 2.3. Functional and Pathway Enrichment Network Analysis of Gene Modules

To determine the gene pathways and biological processes involved in the WGCNA module of interest (the green module in this study, which has the highest correlation with phenotype), the Metascape database (https://www.metascape.org) was used for annotation and visualization [11]. Min overlap ≥ 3 and *P* ≤ 0.01 were considered statistically significant. Membership similarities were detected to distinguish between clusters. Kappa > 0.3 was considered a cluster, and the most statistically significant ones in the cluster were annotated.

### 2.4. Identification of Key Genes in Functional Modules

All genes of the green module were extracted, the included genes were entered into the search tool for retrieval of interacting genes database (https://cn.string-db.org/), and a protein interaction network was visualized by Cytoscape software (version 3.7.1). The degree of connection was calculated for each gene, and the top 10 genes were selected as key genes for subsequent verification.

### 2.5. Verification of the Expression of Target Genes through Experimental Periodontitis Model

In our previous study, the periodontal pathogen *P. gingivalis* (ATCC 33277) was used to establish an experimental periodontitis model in 6-week-old female BABL/c (H-2 dm2) mice. *P. gingivalis* 33277 was cultivated on brain–heart infusion (BHI) agar supplemented with vitamin K1 (10 *μ*g/mL), hemin (0.25%), and sterile defibrinated sheep blood (5%). Bacteria were incubated in an anaerobic atmosphere (Don Whitley Scientific, Shipley, UK) at 37°C. After 7 days, the bacterial colonies were collected and cultured in complete BHI liquid at 37°C for 24 h and then used for oral infection during the logarithmic growth phase.

Animals were fed under standard conditions (humidity: 55–60%, 12 h light/dark cycle, temperature: 20–22°C). After oral bacterial inoculation (10^10^ colony-forming units of *P*. *gingivalis*, once a day for four weeks) or not, the mice were randomly divided into periodontitis and normal control groups. The mice were euthanized by CO2 asphyxiation four weeks after the start of the experiment. The experimental protocol was approved by the Ethics Committee of China Medical University (2019PS119K). The protein was extracted from gingival tissue from each group of mice. Protein expression in the periodontal tissues of periodontitis mice was detected by western blotting.

The extracted protein samples were analyzed using a bicinchoninic acid (BCA) protein assay kit, electrophoresed on 12% SDS-polyacrylamide gels according to their molecular weights, and then transferred to polyvinylidene difluoride (PVDF) membranes. Membranes were blocked with 5% skim milk for 1 h at room temperature. Thereafter, membranes were incubated with rabbit polyclonal anti-FCGR1A (Affinity Biosciences, 1 : 1000) and rabbit polyclonal antitubulin (Affinity Biosciences, 1 : 1000) primary antibodies at 4°C overnight and then incubated with HRP-labeled goat antirabbit IgG secondary antibodies (Affinity Biosciences, 1 : 5000) at 37°C for 1 h. The membranes were visualized using an enhanced chemiluminescence procedure (Enhanced Chemiluminescence Reagent; Millipore, USA).

## 3. Results

### 3.1. Clustering of Samples and Determination of Soft-Thresholding Power

The sample clustering dendrogram and trait heat map of periodontitis samples treated at four different time points are shown in Figure 1(a). According to the standard of a scale-free network, different soft thresholds were obtained through calculations (Figure 1(b)). The correlation coefficient between the logarithm of a node's connectivity [log(*K*)] and the logarithm of the node's probability [log(*P*(*k*))] corresponds to different soft thresholds. Considering the stationarity of the average connection level of the network, we set 14 as the soft threshold, whose correlation coefficient between log(*K*) and log(*P*(*k*)) was close to 0.9, to construct the gene network/module.

### 3.2. Identification of Gene Modules

Through the network construction and initial module division using *β* = 14, we obtained a systematic clustering tree of genes. The dynamic mixed cutting method was used to combine modules with high similarity of characteristic genes. Different colors represent different gene modules: the black module has 219 genes, the blue module has 906, the brown module has 765, the green module has 418, the pink module has 84, and the grey module has 614. Grey represents genes that do not belong to any known module (Figure 2). We finally obtained nine different modules (Figure 3(a)).

### 3.3. Screening of Core Gene Module

Based on the TOM dissimilarity, we used the module eigengene (ME) of each gene module as the overall gene level of the module to correlate with known clinical features. To determine the key modules, correlations between genes and clinical samples in the nine modules were calculated, and the module with the highest correlation was selected as the key module. The results showed that the green module (MEgreen) had the highest negative correlation with disease status (*r* = −0.35, *P* = 0.007), whereas the red module (MEred) was positively correlated with the prognosis of periodontitis treatment (*r* = 0.32, *P* = 0.01) (Figure 3(a)). The clustering analysis indicated that the relevance of green modules is higher (Figure 3(b)). Therefore, genes in the green module at ten weeks postbaseline (four weeks after periodontal treatment) may function as candidate biomarkers for the treatment of periodontal disease. In addition, to explore the coexpression similarity of the nine modules, we calculated the genes of the ten weeks postbaseline group and clustered them according to their correlation. The adjacencies in the ten weeks postbaseline group in the green module network are plotted in a heat map (Figure 3(c)). In the green module of the ten weeks postbaseline group, the correlation between gene significance (GS) and module membership was significant (cor = 0.44, *P* < 0.01) (Figure 3(d)).

### 3.4. Pathway and Process Enrichment Analyses

All genes in the green module of the ten weeks postbaseline group were used as enrichment backgrounds. Pathway and process enrichment analyses showed that most of the biological processes (BP) of the genes were associated with a term related to myeloid leukocyte activation. These genes were also found to be involved in the regulation of cell activation, cytokine production, regulation of leukocyte-mediated immunity, cytokine-mediated signaling pathways, immune response-regulating signaling pathways, regulation of innate immune responses, negative regulation of immune system processes, response to bacteria, regulation of vesicle-mediated transport, regulation of neutrophil activation, chemotaxis, superoxide metabolic processes, cellular regulation of secretion, leukocyte differentiation, negative regulation of the defense response, and macrophage activation (Figure 4(a)). Each node represents an enriched term, and the color of the node indicates the cluster to which it belongs (Figure 4(b)). Terms in the same cluster are closer to and more closely related to each other. The gene set obtained in this study was enriched for immune-related pathways. The green module of the ten weeks past-baseline group has biological significance.

### 3.5. Protein-Protein Interaction (PPI) Enrichment Network Construction and Key Gene Verification

In the visualized protein-protein interaction expression network, parts of networks with highly connected areas have a higher probability of participating in biological regulation, whereas lightly connected nodes will not play a key role in the integrity of the whole network (Figure 5). According to the sort node degree, we screened the top ten genes as candidate genes for further analysis. These were *ARRB2*, *BIRC3*, *CD14*, *DYNLL1*, *FCER1G*, *FCGR1A*, *FCGR2B*, *FGR*, *HCK*, and *PRKCD*. As these genes are closely linked and are at the hub of the PPI network, they are expected to become targets for periodontitis treatment.

### 3.6. Expression and Validation of Key Genes

The expression status of candidate genes was validated in GSE43525, and differentially expressed genes (DEG) were screened in the green module with the cutoff at *P* < 0.05. The candidate genes obtained from the PPI network were validated in the normal and refractory periodontitis samples (Figure 6(a)). As shown in the boxplot, the expression of *CD14*, *FCGR1A*, *DYNLL1*, and *FCGR2B* correlated with disease status; therefore, these data suggest that these key genes may be important targets for the treatment of periodontal disease. We screened 921 DEG from GSE43525 and 418 DEG from the green module of GSE6751. Furthermore, a Venn diagram was used to analyze common DEGs between the GSE43525 and GSE6751 green module datasets (Figure 6(b)), and seven genes were identified: *AMICA1*, *KDELR1*, *DHRS7B*, *LMNB1*, *CTSA*, *S100A12*, and *FCGR1A*.

### 3.7. Western Blotting to Verify the Expression of *FCGR1A* in Experimental Periodontitis Model

Western blot analyses showed an increasing trend with the expression level of FCGR1A protein in periodontal tissues of experimental periodontitis mice compared to normal mice; however, the difference was not statistically significant (Figure 7).

## 4. Discussion

Globally, the prevalence of periodontal disease increases with age from adolescents to adults and older population. Moreover, the low- and middle-income countries had higher occurrence of periodontal disease than high-income countries [12]. The epidemiologic and a large number of clinical and basic studies have found that periodontal health impacts systemic diseases (such as diabetes, metabolic syndrome, obesity, eating disorders, liver disease, cardiovascular disease, Alzheimer disease, rheumatoid arthritis, adverse pregnancy outcomes, and cancer), and vice versa [13]. The prevalence of serious systemic diseases continues to increase and occur in younger patients. Systemic diseases associated with periodontal disease have no specific treatment target; therefore, identification of these therapeutic targets is of great importance. In this study, genes in the peripheral blood microarray dataset GSE6751, consisting of patients with periodontitis, were clustered using bioinformatic methods. The association between the gene modules and specific phenotypes was analyzed using WGCNA. We found that genes with DEG at one month after periodontal treatment (ten weeks postbaseline) exhibited significant alterations in gene expression in the green module. According to pathway and process enrichment analyses, genes involved in immune regulation and lymphocyte-mediated endogenous immune responses, such as regulation of innate immune response, regulation of neutrophil activation, cytokine-mediated signaling pathway, and macrophage activation, play an important role in the treatment of periodontitis. Our group has conducted several previous studies using animal models and found an imbalance in the regulatory function of immune cells in bacterial-induced periodontitis, as well as an imbalance in CD4^+^ or CD8^+^ Treg infiltration and Th17 expression in gingival local tissue, peripheral lymphoid tissue, and spleen in mice during periodontitis [14, 15]. When the lesion was established, the number of infiltrating B lymphocytes in periodontal lesion tissue was significantly higher than the number of T cells; furthermore, the ability of memory B cells to express RANKL was also significantly higher than that of T cells [16, 17]. Moreover, proinflammatory cytokines (IL-1, IL-6, and TNF families), T cell subset-related cytokines (IL-12, IFN-*γ*, IL-4, IL-23, IL-17, TGF-*β*, and IL-10 family), and B cell-related cytokines (IL-10 family) modulate the local host immune responses [18, 19]. Our previous studies indirectly verified our pathway and process enrichment analyses, indicating that periodontal disease develops because of immune cell imbalances, lymphocyte-mediated immune responses, and cytokine-mediated signaling pathways.

Based on the interactive relationship between different genes with the highest connectivity, we identified *ARRB2*, *BIRC3*, *CD14*, *DYNLL1*, *FCER1G*, *FCGR1A*, *FCGR2B*, *FGR*, *HCK*, and *PRKCD* as candidate genes. We used GSE43525 to verify these 10 candidate genes and found a difference in *FCGR1A* expression in refractory periodontitis. Moreover, *FCGR1A* exists at the intersection of Venn diagrams; therefore, we speculated that *FCGR1A* may be a candidate target gene in chronic periodontitis refractory to conventional therapy.

*FCGR1A*, also known as CD64, is an IgG receptor with a high affinity that generally appears in the early stages of the inflammatory response. As one of the receptors of the IgG Fc fragment, CD64 can recognize immunoglobulin and has a high affinity for IgG monomers (IgG1 and IgG3). Under normal physiological conditions, CD64 is constitutively expressed on macrophages, monocytes, and eosinophils and, to a lesser extent, on resting neutrophils. However, in a state of infection or inflammation, CD64 expression on the surface of neutrophils can be increased rapidly, and the expression can be multiplied 5–10 times. Such engagement is stable in the body and represents a reliable biomarker for the early diagnosis of bacterial infection [20]. In the initiation and maintenance of a series of chronic diseases, CD64 is considered as a bridge connecting humoral and cellular immunity. It affects phagocytosis, clearance of immune complexes (such as inhibition of IFN-*γ* and TLR4 signaling), antigen presentation, and stimulation of the release of inflammatory mediators [21–23]. CD64 engagement also regulates immune inflammation by promoting NF-*κ*B regulation of NLRP3 inflammasome signaling [24, 25]. In the gingival tissue of patients with chronic periodontitis, the expression of MMP-12 in CD64-derived monocytes increased significantly, and the expression of surface costimulatory molecule, CD200R, decreased, resulting in irreversible tissue decline and immune activation disorders [26]. CD64 is considered to have significant clinical potential in resolving chronic inflammation driven by M1-type dysregulated macrophages [27, 28].

## 5. Conclusion

In summary, we constructed a coexpression network using WGCNA, detected gene modules, and identified 10 candidate genes for periodontal comprehensive therapy. We used the GSE43525 database to verify candidate genes and confirm *FCGR1A* (CD64) as a key gene in the development of periodontitis. These findings were drawn using bioinformatics approaches and validated by experimental periodontitis model. We expect that *FCGR1A* (CD64) may be a potential target for evaluating the prognosis of comprehensive periodontal therapy.

Nonetheless, this study has limitations that could to be addressed in future research. Currently, our focus is on using bioinformatics to analyze the results of published studies. However, the patient sample size of these studies is limited. Increase in research will increase the number of expression databases available in the Gene Expression Omnibus. Additionally, the potential target gene screened in this study has only been confirmed in animal models of periodontitis. In the future, we aim to reevaluate the expression of *FCGR1A* (CD64) in human periodontal ligament cells or tissues.

## Figures and Tables

**Figure 1:** Clustering of samples and determination of soft-thresholding power. (a) The clustering was based on the expression data of GSE6751, which contained 59 samples of blood at four time points: 15 samples at 1 week prior to periodontal treatment, 14 samples at treatment initiation, 15 samples at 6 weeks postbaseline, and 15 samples at 10 weeks postbaseline. (b) Analysis of the scale-free fit index for various soft-thresholding powers. (c) Analysis of the mean connectivity for various soft-thresholding powers.

**Figure 2:** Clustering dendrograms and modules identified by WGCNA. (a) Heat map depicts the topological overlap matrix (TOM) of genes selected for weighted coexpression network analysis. Blue represents lower overlap, and red represents higher overlap. (b) Each branch in the figure represents one gene, and each color represents a module in the constructed gene coexpression network by WGCNA.

**Figure 3:** (a) Heat map of the correlation between module eigengenes and the disease status of periodontitis. The turquoise module was the most positively correlated with status, and the green module was the most negatively correlated with status. (b) Hierarchical clustering of module hub genes that summarizes the modules yielded in the clustering analysis. (c) Heat map of the adjacencies of the 10 weeks postbaseline group in the green module network. (d) Scatter plot of module member ship (MM) vs. gene significance (GS) in the green module. Cor represents the absolute correlation coefficient between MM and GS, and *P* is the significance evaluation.

**Figure 4:** Pathways and process enrichment analyses. (a) The GO enriched terms colored by the *P* value. (b) Network of enriched terms colored by cluster identity, where nodes that share the same cluster identity are typically close to each other. Each term is represented by a circle node, and its color represents its cluster identity.

**Figure 5:** The protein-protein interaction enrichment clusters have nodes colored according to the *P* value. Each point represents a gene, and the edges connecting genes represent the interactions between genes. The darker the color and the node size, the higher the degree of connectivity of the genes.

**Figure 6:** (a) Boxplot of the key candidate genes in expression level in GSE6751 with four groups (^∗^*P* < 0.05). (b) Boxplot of the key candidate genes in expression level between control and refractory periodontitis (^∗^*P* < 0.05). (c). Different express genes were selected by Venn diagrams.

**Figure 7:** Protein expression of FCGR1A in periodontal tissues was analyzed by Western blot.

## Data Availability

All data included in this study are available upon request by contact with the corresponding author.
